# The Effect of lncRNA-PVT1 on Liver Cancer Rats by Regulating the Expression of MMP9

**DOI:** 10.1155/2022/4126839

**Published:** 2022-09-17

**Authors:** Bin Lu, Min Cheng, Tao Wang

**Affiliations:** Department of Hepatological Surgery, Chaohu Hospital of Anhui Medical University, Chaohu, Anhui, China

## Abstract

As a malignant tumor, liver cancer has a high lethality rate. The research on the pathogenesis of liver cancer is the key to the treatment of liver cancer. The latest research claims that lncRNA-PVT1 as a tumor gene participates in the generation and development of tumors by regulating matrix metalloproteinase MMP9. The purpose of this article is to explore the specific effect and mechanism of lncRNA-PVT1 on liver cancer rats by regulating the expression of MMP9. In this article, 50 rats are used as experimental subjects, the rats are divided into control group and observation group, and the liver cancer cell line HepG2 is cultured. The transplanted tumor liver cancer model was constructed by transfection of hair, the expression of lncRNA-PVT1 in the observation group was reduced by knockdown method, the expression levels and changes of lncRNA-PVT1 and MMP9 in the two groups were detected by PCR fluorescence method, and the difference between lncRNA-PVT1 and MMP9 was analyzed. The MTT method was used to detect the proliferation, migration, and invasion capabilities of the two groups of liver cancer cells (LCC) and to explore the effect of lncRNA-PVT1 on rat LCC by regulating the expression of MMP9. The results of the study showed that after knocking down the expression of lncRNA-PVT1 in the observation group, the expression of MMP9 also decreased. At the same time, the migration rate of LCC HepG2 decreased by 27.4%, the level of invasion ability decreased by 21.6%, and the proliferation rate of LCC decreased by 17.8%. Therefore, it can be seen that lncRNA-PVT1 plays a positive regulatory role on the expression of MMP9, and the expression of MMP9 promotes the proliferation, migration, and invasion of rat LCC.

## 1. Introduction

Liver cancer has always been the most common disease among adult patients with malignancies in China, although the early treatment and rehabilitation techniques for adult liver cancer have been continuously improved, such as surgical liver resection, liver transplantation, radiotherapy, and chemotherapy. However, the overall 5-year survival rate of many patients with advanced liver cancer has not improved significantly. One of the important reasons for the high mortality and poor prognosis of liver cancer is that the main molecular immune mechanism of the early occurrence and development of liver cancer is still poorly understood.

Long-chain nonlinear coding RNA lncRNA coding is a hot spot in medical research in recent years. Current studies have found that lncRNA still has important cell biology coding functions, such as regulating human cell benign proliferation, cell cycle, cell differentiation, and cell benign apoptosis [1]. In addition, the abnormal cell expression of lncRNA is closely related to the treatment of various human diseases, especially in the treatment of malignant tumors [2]. As a type of tumor molecular gene, PVT1 is abnormally expressed in multiple types of tumors and can therefore simultaneously regulate multiple tumors. This article focuses on the correlation between lncRNA-PVT1 and MMP9 [3].

In order to explore the specific effect and mechanism of lncRNA-PVT1 on liver cancer rats by regulating the expression of MMP9, a large number of related materials were consulted. Among them, Wu et al. introduced the pathogenesis of liver cancer in detail and analyzed several main common treatment methods that are still commonly used in the treatment of chronic liver cancer in China; the main methods include new hepatitis B early surgical treatment combined with treatment, radiotherapy combination of chemotherapy, and other hepatitis B drug therapy [4]. Xiong et al. pointed out in his article that most liver cancer patients are carriers of hepatitis B virus and discussed the current status of liver cancer research in China, pointing out that if liver cancer cannot be detected early and treated in time, it will bring a high mortality rate, and emphasized cirrhosis and liver ascites are the clinical manifestations of advanced liver cancer [5]. In the article, Iden et al. introduced the relationship between long-chain noncoding lncRNA and tumors, discussed the mechanism of lncRNA in the treatment of liver cancer, and emphasized that PVT1, as a downstream factor of tumor cells, promotes the formation and development of liver cancer [6]. Lu et al. found through research that there is a close relationship between the expression of matrix metalloproteinase MMP9 and tumor cells, pointing out that overexpression of MMP9 is not good for the treatment of liver cancer, and proved that MMP9 is an oncogene [7]. Through research, Li et al. found that lncRNA-PVT1 has a certain effect on the changes of LCC by regulating the expression of MMP9, and he pointed out that lncRNA-PVT1 can promote the expression of MMP9, thereby affecting the proliferation, migration, and invasion ability of LCC [8].

In the study of the specific effect and mechanism of lncRNA-PVT1 on liver cancer rats by regulating the expression of MMP9, this article summarizes and analyzes the research experience and results of a large number of predecessors. In addition, this article has made some innovations in research content and detection methods. There are two specific innovations as follows: first, this article uses tumor cell transfection to create a rat liver cancer animal model, uses a multicomponent statistical data analysis method collected by data analysis software, and uses PSPY software to carry out liver cancer cell transfection. The statistical data collection and analysis of the detection results of changes in various indicators greatly improves the accuracy of the research results. Second, firstly, it focused on the direct relationship between the abnormal gene expression of lncRNA-pvt1 in malignant liver cancer early tumor cell tissue production and the early clinical pathological response characteristics of liver cancer tumor cells and then focused on the expression of this gene in liver cancer. The cell generation function of tumor patients has a direct impact on the sensitivity of liver cancer chemotherapy drugs. Finally, the prognostic value of lncRNAPVT1 by regulating the expression of MMP9 in patients with malignant tumors was evaluated.

## 2. Relevant Experiments to Construct Rat Liver Cancer Model

### 2.1. Rat Selection

In this experiment, 50 male SD rats were selected as the research objects, with an average age of 8 to 12 months and a weight of (250 ± 3.0) g. The laboratory that has been disinfected and pollution-free was selected as the experimental site, and the laboratory temperature was 16-24°C, the moisture in the air is about 16.3-20.8%, the laboratory maintains ventilation to ensure sufficient oxygen content in the air and raises them in cages according to the national standard whistle-dent animal feeding specifications. Check the health of the rats before the experiment rats with abnormal health.

### 2.2. Experiment Related Equipment

The main equipment used in this experimental research is liver cancer cell line HepG2, PCR fluorescence detector, SKB-500 type microplate reader, western blot electrophoresis equipment, flow cytometer, and section paraffin embedding machine. ACL-V8 animal ventilator, POWER-8 model physiological signal acquisition instrument, LEICB-218 slicer, BX230 electron optical microscope, image analyzer (Jiangsu Zhongdu Analytical Instrument Co, Ltd.), fluorescence display, automatic blood analyzer, BCL-210A Rongcheng water tank (Jiangsu Branch Thai Electric Co., Ltd.), and electronic balances are produced by Stayer Company. The relevant reagents used in this experiment are shown in Table 1. The qPCR primer sequences that were used were lncRNA PVT1 forward primer 5′-TGAGAACTGTCCTTACGTGACC-3′, reverse primer 5′-AGAGCACCAAGACTGGCTCT-3′, GAPDH forward primer 5′-GGTTGTCTCCTGCGACTTCA-3′, and reverse primer 5′-TGGTCCAGGGTTTCTTACTCC-3′, MMP9 forward primer 5′-GAACTTTGACAGCGACAAGAAG-3′, and reverse primer 5′-CGGCACTGAGGAATGATCTAA-3′.

### 2.3. Hepatoma Cell Culture

A cell rpm-1640 medium containing 10% FBS and 1% penicillin was used to culture normal hepatocarcinomatous cells hepg2, bel-742, and normal adult hepatocyte culture strain l02 cells. Normal culture conditions are culture in a 10% co. incubator, the temperature is constant at 30°C, and saturated humidity. The normal hepatocarcinomatous cells hepg2 were cultured to the logarithmic growth phase and carefully observed under a microscope, and the digestive juice can be passaged for subsequent experiments. Cultivation method after normal LCC is digested, hepg2 is covered to 70~80% of the bottom of the penicillin culture flask, aspirate the old penicillin culture medium, rinse the pbs with water, and add a little penicillin combined. Digestion solution, shake the penicillin streptomycin culture flask gently to make the combined digestion solution evenly flow over the surface of LCC, and place it in a new incubator. After 1 min, observe carefully under a light microscope, and see that the cell gap in the culture medium gradually increases and when the cells become rounded, a small amount of deem joint culture medium is added, then the joint digestion is terminated, and the cells are gently blown with a pipette. Transfer the supernatant to the cell centrifugation master, centrifuge at 1000 r/min for 5 min, aspirate the cell supernatant and then wash it twice with soap pbs, continue centrifugation at 1000 r/min for 5 min, and aspirate and discard the clear liquid pbs in the cell from the tube. After filtering, add it to PCD and reset the culture solution to form a suspended cell. After 1 : 2 or 1 : 3 passage, place it in a small culture room incubator with a normal constant temperature and then perform the second time to cultivate.

### 2.4. Establishment of Rat Liver Cancer Animal Model by Transfection Method

Dilute the hepg2 in the logarithmic growth phase to ix107 cells/ml, inoculate it in an 8-well plate, and culture the cells to a confluency of 70-80% for cell transfection. First use the diluted serum-free mem medium to dilute the liposomes and the fragments and carriers of each group, and then gently mix the diluted equal volume of liposomes, the carriers and fragments of each group, and incubate for 30 minutes at room temperature. The mixture was dropped into the already cultured liposomes and hepg2 cells, mixed gently, placed in a 34°C, 10% co2 incubator for 5 hours, replaced with rpmi-1640 complete medium, transfected for 48 hours, and the liver cancer. The cell line was injected into the rat with a syringe to verify the transfection effect. One week later, observe whether the rat liver cancer tumor cells are formed to determine whether the modeling is successful.

### 2.5. Detection of MMP9 Expression Level

Collect normal liver cells and LCC in each group, extract total RNA from the cells according to the requirements of the MMP9 extraction kit, and store them at -60°C. When the fusion rate of LCC is about 80%, PCR fluorescence method is used to detect the level of MMP9 expression of related molecules in LCC.

### 2.6. Detection of Proliferation, Migration, and Invasion Ability of LCC

Detection of cell migration ability: each group of HepG2 cells after cell transcription infection is cultured to normal logarithmic growth phase, the cells are collected, and diluted protein-free serum rpim-1640 medium containing 1% BSA is added to the diluted cells. The concentration is 2.5 × 105 pcs/ml. Put the upper chamber cells into the lower chamber and place them in a 37°C 5% CO_2_ incubator for 24 hours. Use a cotton swab to gently wipe off the fixed and migrated cells in the upper chamber. Ice formaldehyde is used as the fixed and migrated cells, stained with crystal violet, and observe the cell count under microscope.

Invasion ability test: all reagents and other test equipment are precooled on ice, put the cells in the trial chamber and place in a 24-well plate, and evenly smear 80 *μ*L (0.5 g/l) of glue on the inner membrane of the chamber, starting at 33°C incubate for 15 min to make the gel completely solidify. After digestion, centrifugation, and counting to take out the cells, the cells were diluted with nonfetal bovine serum medium according to 2.5 × 10^5^/L to make a nonfetal cell digestion suspension. According to 200 *μ*L per well, add the suspension for cell digestion from the lower chamber to the upper chamber of the trill, and at the same time, add 20% fetal calf serum +300 all of the medium to the lower chamber of the trill, put it in the initial incubator at 34°C for culture, and formaldehyde fixation, stain with crystal violet for 20 minutes, and then gently wipe the cells on the chamber membrane with a cotton swab. Cell count under a high-power field microscope 4 cells that penetrate and filter the chamber membrane under a high-power field microscope are counted.

Proliferation ability detection: MT method is used to detect cell proliferation. The lncRNA, which is the most effective inhibitor of PVTI expression, was screened and transfected into HepG2 cells of liver cancer. The HepG2 cells in logarithmic growth phase were used for logarithmic growth phase and seeded into 96-well plates, and routine cells were performed four times in each well. After culturing for 24, 48, and 72 hours, discard it to remove the logarithmic medium in the growth phase. After adding mt each time, add mt repeatedly and continue to perform routine cell culture per well for 3 hours. After adding one mt, it can make demos cell lysis, using automatic cell fluorescence emission microplate reader to continuously detect the total absorption fluorescence of granulocytes per well (a value). The cell absorption fluorescence value of each well can be repeated continuously for 4 times.

## 3. The Effect of lncRNA-PVT1 Regulating the Expression of MMP9 on LCC

### 3.1. Analysis of the Effect of lncRNA-PVT1 on the Proliferation, Invasion, and Migration of LCC by Regulating the Expression of MMP9

The results of the study showed that the expression of lncRNA-PVT1 in the control group was significantly lower than that of the observation group, and the expression of MMP9 in the observation group was higher than that of the control group. After successful transplantation of LCC, the expression of lncRNA-PVT1 in the observation group increased significantly and was higher than that of the control group, indicating that LCC induced an upregulation of lncRNA-PVT1 expression. Studies have found that lncRNA-PVT1 can regulate the expression level of MMP9 in rat LCC. The effects of the successful establishment of rat liver cancer animal model and the reduction of lncRNA-PVT1 expression on the expression level of MMP9 are as shown in Table 2.

The results showed that the expression of MMP9 after knockdown of lncRNA-PVT1 was significantly reduced, and the proliferation of LCC was significantly reduced (*P* < 0.05), while the proliferation of LCC transfected with lncRNA-PVT1 was significantly higher than that of the observation group (*P* < 0.05). It can be seen that reducing lncRNA-PVT1 can reduce the expression of MMP9, thereby inhibiting the proliferation activity of LCC. The research results show that lncRNA-PVT1 can affect the proliferation of rat LCC by regulating the expression of MMP9. The relevant data are shown in Figure 1.

From the data in Figure 1, it can be seen that lncRNA-PVT1 can affect rat LCC by regulating the expression of MMP9, and regulating the expression of MMP9 by knocking down lncRNA-PVT1 can reduce the proliferation rate of LCC by 17.8%.

After transfection of lncRNA-PVT1 to reduce the expression of MMP9, the migration ability of HepG2 cells was significantly lower than that of the control group (*P* < 0.05). Upregulating the expression of MMP9 can reverse the inhibitory effect of lncRNA-PVT1 overexpression on LCC, while downregulating its expression can reverse the promotion of MMP9 silencing on gastric cancer cell migration. The study found that the invasion ability of HepG2 cells after upregulating the expression of lncRNA-PVT1 was significantly lower than that of the control group (*P* < 0.05). At the same time, the invasion ability of cells in the control group was significantly lower than that of the observation group (*P* < 0.05), and lncRNA-PVT1 was downregulated. After expression, the migration ability of HepG2 cells is heightened. Downregulating the expression of lncRNA-PVT1 can reverse the promotion of MMP9 overexpression on the invasion of LCC, and downregulating its expression can reverse the promotion of MMP9 silencing on the invasion of gastric cancer cells. The specific data are shown in Figure 2.

It can be seen from the data in Figure 2 that lncRNA-PVT1 can affect the migration and invasion of rat LCC by regulating the expression of MMP9, regulating the expression of MMP9 by knocking down lncRNA-PVT1 can reduce the migration rate of LCC by 27.4%, and the invasion ability the level dropped by 21.6%.

### 3.2. Analysis of the Effect of lncRNA-PVT1 on Tumor Intervention by Regulating the Expression of MMP9

In this paper, QRT-PCR detection found that lncRNA-pvt1 is highly expressed in the study of the relationship between apoptosis of LCC huh7, hepg2, and mmpsmmc-7721, suggesting that lncRNA-pvt1 may be used as a proto-oncogene to control the normal occurrence and development of LCC. The process of apoptosis is an important cell biology inhibitory process, and it plays a vital role in cell suppression in the survival and homeostasis of LCC. MMP9 is an important member of the MMPS protein family and is a key cell regulator and inhibitory factor that controls the apoptosis of LCC. MMP9 protein is located upstream of caspase-3, an apoptotic executor, and can cause caspase-3 activation and induce apoptosis. A large number of studies have confirmed that MMP9 is usually upregulated in tumor cells and is an inhibitor of tumor cell apoptosis, while caspase-3 is a proapoptotic factor. The relevant data are shown in Figure 3.

From the data in Figure 3, it can be seen that knockdown of lncRNA-PVT1 can downregulate the expression of MMP9, thereby promoting the apoptosis of LCC, and regulating the expression of MMP9 by knocking down lncRNA-PVT1 can increase the apoptosis rate of LCC by 16.2%.

In addition, among the four liver cancer cell lines, HepG2 and PaTu8 cells express higher levels of lncRNA-PVT1, while SW1990 has the lowest expression. On the one hand, this paper uses lncRNA-PVT1 specific siRNA to knock out MMP9 to reduce the expression of lncRNA-PVT1 in LCC. On the other hand, the lncRNA-PVT1 expression vector is used herein to increase the expression of MMP9 in LCC. Then through the liver cancer cell function experiment to study the proliferation, apoptosis, erection, invasion, and metastasis of LCC, studies have shown that downregulating lncRNA-PVT1 reduces the proliferation of LCC and promotes apoptosis, thereby accelerating tumor growth. The research results show that lncRNA-PVT1 can interfere with tumor growth rate by regulating the expression of MMP9. The specific data is shown in Figure 4.

It can be seen from Figure 4 that lncRNA-PVT1 can interfere with tumor growth rate by regulating the expression of MMP9, and regulating the expression of MMP9 by knocking down lncRNA-PVT1 can reduce the growth rate of liver cancer tumors by 22.9%.

## 4. Conclusions

As a malignant tumor, liver cancer has a high fatality rate. Research on the pathogenesis of liver cancer and oncogenes is the key to the treatment of liver cancer. The latest research claims that lncRNA-PVT1 as a tumor gene participates in tumor development by regulating matrix metalloproteinase MMP9. Studies have found that knocking down lncRNA-PVT1 in LCC can effectively reduce the expression level of MMP9, proving that lncRNA-PVT1 is an upstream factor of MMP9.

The results of the study show that lncRNA-PVT1 can affect rat LCC by regulating the expression of MMP9, and regulating the expression of MMP9 by knocking down lncRNA-PVT1 can reduce the migration rate of LCC HepG2 by 27.4% and the level of invasion ability by 21.6%. In liver cancer, the cell proliferation rate decreased by 17.8%. Therefore, it can be seen that lncRNA-PVT1 plays a positive regulatory role on the expression of MMP9, and the expression of MMP9 promotes the proliferation, migration, and invasion of rat LCC. Studies have found that knockdown of lncRNA-PVT1 can downregulate the expression of MMP9, and regulating the expression of MMP9 by knocking down lncRNA-PVT1 can increase the apoptosis rate of liver cancer cells by 16.2%.

## 5. Discussion

Hepatitis B virus X protein (HBX) is the only protein expressed in malignantly transformed liver cells and is closely related to the occurrence and development of liver cancer [9, 10]. HBX protein is a basic antiviral immune protein during the growth cycle of virus infection in the body. Its main part is located in the entire cytoplasm, and some smaller parts may be located in the entire nucleus. A type of hepatitis B virus immune x protein in the nucleus usually has a trans-transcription activator effect, which can act on a protein or transcription activator whose binding site is DNA in the nucleus through immune protein-transcription protein interaction. And directly or indirectly act on its gene promoter or gene enhancer to activate it in trans gene [11]. The virus x protein cell in hepatitis B can directly form a virus dimer, docking with acetyl tyrosine kinase (JAK), activating cell JAK, and activated JAK cells can activate f-ap-1, NF-kb-1 to stimulate viral transcriptional activity [12]. This protein also directly binds to many senescent cell-related toxicity inhibitors that can control the survival and normal proliferation of senescent cells. The x protein in the hepatitis B virus directly activates the cell SRC and s/RAS/RAF/ERK (regulation and inhibition of kinases through extracellular transcription signal activity) conversion pathways, which directly leads to the activation of cellular transcriptional trans-inhibition and transcriptional static inhibition of HCC enzymes transformation in the cell [13].

Studies have found that HBVX protein can induce chromosomal changes and microsome formation in liver cells. The number of microsomes in hepg2 cells transfected with HBVX protein increased three times faster than that in the control group of cells with HBVX protein transfected [14]. The hepatitis B virus X protein can promote the formation of abnormal central cells and multipolar spindles, increase the centrosome to cause abnormal mitosis, the chromosomes represented increase the possibility of errors, and the hepatitis B virus X protein in the cytoplasm can CRML (able to interact with Da/P enzyme). Isolate the output of nuclear receptor 1 (CRML), induce nuclear factor (NF-KB) approval, use cell CRML mutation to inhibit cytokine to participate in the treatment of tumor cells are observed and detected in tumor cells. The number has increased significantly, and the x protein activity mutation inhibitor in some hepatitis B late virus has not been observed and detected, suggesting that cell CRML is actively involved in processing to maintain the structural integrity of the cell centrosome, hepatitis B late virus. The activity of the x-protein mutation inhibitor CRML in the protein cannot destroy the structural integrity of the entire genome, which greatly increases the potential death risk of patients suffering from chronic liver cancer. In the early stage of hepatitis B virus cell X protein has an immunomodulatory effect on the rapid apoptosis and normal proliferation of prokaryotic cells. It is a multifunctional immune protein. ACTS protein can be used in different immune targets (including transcriptional immune factors, cellular immune kinases, and mitochondrial immune proteins); it can simultaneously regulate the normal proliferation and apoptosis of early tumor prokaryotic cells of hepatocellular carcinoma [15].

The interaction between early hepatitis B virus and methyl p53 has a certain inhibitory effect on the malignant proliferation and apoptosis of early tumor epithelial cells of hepatitis B [16]. Hepatitis B late virus inhibits the enzyme of the x protein and the terminal binding region of the c cell. Cells can directly bind to the wild-type virus p53 protein in the virus cytoplasmic structure and thereby prevent their cells from entering the virus nucleus, thereby producing cell transcription that inhibits virus p53, thereby produce influence pnwtp53 to prevent the growth of abnormal virus nuclei, and thereby promote the transcription ability of PNDNA repair. In the presence of a virus greater than p53 infection, hepatitis B bacterial virus cell x protein growth-inducing enzyme and p21t protein lead to growth arrest in G1 phase, leading to early apoptosis of virus cells, thereby effectively promoting the early acute hepatitis B cell virus infection sustainable development [17]. In the case that the virus lacks transcription through p53, the immunosuppressive effect of the x protein in the hepatitis B virus on the transcription through p2141 can promote the rapid differentiation and proliferation of those proto carcinoma cells that are not under immune control, thereby serving as proto carcinoma cells. Mutations in genes or genes that are tumor immunosuppressive agents accumulate and eventually lead to the occurrence of liver cancer [18]. The decrease of P53 activity leads to defects in DNA repair function, which enables damaged cells to enter the DNA synthesis and division stage through the G and G stages smoothly, and obtains a new transformed phenotype. When the tumor progresses to an advanced stage, the hepatitis B virus X protein can promote the proliferation of malignant transformed cells and accelerate the development of the tumor [19, 20].

According to the relative sequence position of lncRNA in the genomic sequence of each type of protein gene coding, lncRNA can be divided into 5 categories at present. The first method is to encode the sense gene lncRNA, which is usually transcribed from a sense link that encodes the sense gene in a proteome. The second type is antisense lncRNA transcription from the antisense strand of protein coding genes. The third type is bidirectional, which can be simultaneously transcribed in the same or opposite direction as the transcription direction of adjacent mRNA. The fourth is genomics, which is transcribed from the space between two protein-coding genes. The fifth type is lncRNA, which is transcribed from the intron region of the gene encoding it [21]. lncRNA is distributed in the cytoplasm, nucleus, and organelles, with complex and diverse functions. They can regulate epigenetic, transcription, and posttranscriptional gene expression and are widely involved in almost all physiological and pathological processes of the human body [22].

The complex and precise gene regulation mechanism function of lncRNA greatly explains the expression and complexity of daily life genes and helps people to understand the genetic complexity and complexity of daily life from the perspective of gene expression and the complexity of regulating gene networks. Development has opened up new scientific horizons. Existing studies have shown that lncRNA can participate in a series of cell biology processes, such as cell proliferation, apoptosis, invasion, migration, cell cycle, and cell differentiation [23, 24]. Malat-1 expression is upregulated in liver cancer cell lines and 88 clinical tissue samples, and malat-1 silencing may inhibit the proliferation, migration, and invasion of normal liver cancer tumor cells. Therefore, malat-1 may be considered as a predictor of normal liver a new type of liver cancer tumor biochemical marker for the recurrence of liver cancer malignant tumor after cell transplantation. lncRNA is highly expressed in various malignant tumors and is closely related to the poor prognosis [25]. Through analysis and detection of clinical liver cell tissue samples from patients with normal liver cancer and malignant tumors and normal liver cell tissue samples, the clinical tumor expression pathological diagnosis level of hot air in patients, the clinical tumor expression pathological diagnosis level of hot air in liver cancer patients and clinical tumors in liver cancer patients, and the internal correlation between the pathological diagnosis parameters, it is found that the tumor expression of hotwire in liver cancer patients is closely related to the differentiation, metastasis, and early tumorigenesis of liver cancer. Recurrence is an important biomarker for early diagnosis of liver cancer and other malignant tumors [26].

lncRNA and signal transduction have brought new hopes and breakthroughs in leading and treating liver diseases. Studies have shown that the mechanism of lncRNA on liver disease is the result of a combination of multiple factors. lncRNA can not only interfere with the expression of downstream genes but also affect the biphasic regulation of TGF-cells in tumors [27]. In the early stages of tumors, TGF-polymers exert antitumor effects by inducing cell cycle arrest and apoptosis. Studies have reported that TGF-TGF-small molecules interact with lncRNA to promote the occurrence and development of liver cancer. Studies have found that TGF-small molecules induce the upregulation of lncRNA-ATB expression in liver cancer. lncRNA-ATB then competitively binds to miR-200 family members, upregulates the expression of ZEB1 and ZEB2 in the E-box-binding zinc finger protein (ZEB) family, and ultimately promotes the occurrence of EMT of LCC and gains invasive ability [28]. Further research found that lncRNA may act as an upstream activator of TGF-case1, upregulate TGF-case1 signal transduction, promote the invasion and migration of LCC, and aggravate the development of liver cancer.

The results of the study showed that after knocking down the expression of lncRNA-PVT1 in the observation group, the expression of MMP9 also decreased. At the same time, the migration rate of LCC HepG2 decreased by 27.4%, the level of invasion ability decreased by 21.6%, and the proliferation rate of LCC decreased by 17.8%. Therefore, it can be seen that lncRNA-PVT1 plays a positive regulatory role on the expression of MMP9, and the expression of MMP9 promotes the proliferation, migration, and invasion of rat LCC.

## Figures and Tables

**Figure 1:** The effect of lncRNA-PVT1 on the proliferation of rat LCC by regulating the expression of MMP9.

**Figure 2:** The effect of lncRNA-PVT1 on the migration and invasion of rat LCC by regulating the expression of MMP9.

**Figure 3:** Knockdown of lncRNA-PVT1 and downregulation of MMP9 expression affects the apoptosis rate of hepatocellular carcinoma cells.

**Figure 4:** The effect of lncRNA-PVT1 on tumor growth rate by regulating the expression of MMP9.

**Table 1:** Related reagents used in this experiment.

Group	Usage amount	Source
Running buffer	500 ml	Japan Sanyo Corporation
Agar powder	300 ml	American Bio-Rad
DNA marker	240 ml	Jimi Electronic Technology Company
Cell counting kit-8	600 ml	Japan Associates
Hydrochloric acid	450 ml	Gaohu Chemical Enterprise
Sulfuric acid	300 mg	Japan Sanwa Kimono
Sodium chloride	280 ml	American SGH
Trypsin	520 ml	Gibco Corporation United States
Matrigel Matrigel	1200 ml	Taker (Dalian) Co., Ltd.

**Table 2:** The effect of reducing the expression of lncRNA-PVT1 on the expression level of MMP9.

Group	lncRNA-PVT1	MMP9	After knocking down	Before knocking down
Control group	76.3 ± 3.68	85.3 ± 4.15	107.6 ± 5.58	158.4 ± 6.36
Observation group	72.4 ± 3.92	91.6 ± 5.21	123.2 ± 4.95	165.3 ± 5.75
*T*	12.36	11.47	10.15	13.28

## Data Availability

All data, models, and code generated or used during the study appear in the submitted article.
